The article "Clinical Study on Effect of Solution Focused Approach on the Complications, Pain, Sleep, and Quality of Life in Patients with Hepatocellular Carcinoma Undergoing TACE" was retracted in 2023. Reasons: unreliable results or conclusions; concerns about the data; concerns about the peer review; concerns about the citations.

# Clinical Study on Effect of Solution Focused Approach on the Complications, Pain, Sleep, and Quality of Life in Patients with Hepatocellular Carcinoma Undergoing TACE

**DOI:** 10.1155/2021/5068228

**Published:** 2021-09-15

**Authors:** Chunjie Ma, Yuexian Ma, Sidi Lu, Dan Li, Yan Wang, Yingxuan Xu, Tianyu Zhang, Youli Du, Lulu Wang

**Affiliations:** ^1^Department of CT, The Second Affiliated Hospital of Qiqihar Medical University, Qiqihar, Heilongjiang 161006, China; ^2^Department of Nursing, The Second Affiliated Hospital of Qiqihar Medical University, Qiqihar, Heilongjiang 161006, China; ^3^Department of Gastroenterology, The Second Affiliated Hospital of Qiqihar Medical University, Qiqihar, Heilongjiang 161006, China; ^4^Department of Intervention, The Second Affiliated Hospital of Qiqihar Medical University, Qiqihar, Heilongjiang 161006, China; ^5^Department of Anatomy, Qiqihar Medical University, Qiqihar, Heilongjiang 161006, China

## Abstract

**Objective:**

The objective of this study is to explore the effect of solution focused approach (SFA) on the complications, pain, sleep, and quality of life in patients with hepatocellular carcinoma undergoing transcatheter arterial chemoembolization (TACE).

**Methods:**

Total of 106 patients with hepatocellular carcinoma who underwent TACE in our hospital from July 2019 to June 2020 were selected. According to the admission time, they were divided into the control group (*n* = 53) and the observation group (*n* = 53). The control group implemented routine nursing intervention, and the observation group implemented SFA on the basis of the control group. The clinical data, complications, pain, sleep status, and quality of life scores were compared between the two groups.

**Results:**

The total incidence of complications in the observation group (16.98%) was lower than that in the control group (33.96%) (*P* < 0.05). There was no significant difference in the score of pain perception between the two groups (*P* > 0.05). The scores of sleep status in the observation group were lower than those in the control group (*P* < 0.05). The quality of life scores in the observation group was higher than that in the control group (*P* < 0.05).

**Conclusion:**

SFA can effectively reduce the complications, relieve pain, improve sleep status, and improve the quality of life in patients with hepatocellular carcinoma undergoing TACE.

## 1. Introduction

Hepatocellular carcinoma is the cancer that originates from hepatocyte or biliary tract cell. Patients with hepatocellular carcinoma generally have no obvious symptoms in the early stage. With the development of the disease, the symptoms of hepatalgia, hypodynamia, anorexia, and ventosity may appear, which seriously affect the life safety of patients [1, 2]. The survey showed that in 2020, hepatocellular carcinoma ranks sixth in the morbidity and ranks third in the mortality of cancers in the world, and the number of patient increases year by year [3]. Nowadays, transcatheter arterial chemoembolization (TACE) is the effective method to treat hepatocellular carcinoma. It is easy to be operated, less traumatic, economical, adaptive to a wide range, and able to prolong the survival time of patients with effective outcome [4, 5]. However, TACE generally brings patients physical discomfort of different degrees which brings negative emotions that increase the psychological pressure of patients, influence the prognosis in a negative way, and reduce the quality of life of patients [6, 7]. Therefore, it is important to take scientifically reasonable nursing towards patients with hepatocellular carcinoma undergoing TACE.

At present, people's expectation towards medical service is becoming higher and the nursing working mode is changing. The solution focused approach (SFA) is the intervening model that works through guiding individual to find problems and set goals and then solves the problems focusing on the positive aspects of the individual. It has the characteristics of simple, effective, and affordable and has played a key role in a variety of diseases such as overweight and diabetes [8, 9]. The SFA can fully explore the potential of individuals by guiding individuals to formulate scientific and feasible plans, stimulate their subjective initiative, and enhance their ability to manage themselves correctly so as to solve the current problems and improve the living standards of individuals. In addition, the SFA can not only intervene with the physical state of the body but also affect the mental health of the people. This model can effectively mobilize the enthusiasm of individuals and improve the efficiency of the self-management and the meaning of life, reduce negative emotions, and enable people to establish good beliefs and improve the psychological resilience of individuals, which is a promising intervention approach.

The SFA plays an important role in clinical treatment at home and abroad. However, research on the application effect of SFA in patients with hepatocellular carcinoma undergoing TACE is relatively rare. Our physicians apply SFA to patients with hepatocellular carcinoma undergoing TACE through the summary of clinical experience and the inquiry of the literature. The paper is aimed to explore the effect of SFA on the complications, pain, sleep, and quality of life of patients with hepatocellular carcinoma undergoing TACE.

## 2. Materials and Methods

### 2.1. General Information

Total of 106 patients with hepatocellular carcinoma who underwent TACE in our hospital from July 2019 to June 2020 were selected. There were 60 males and 46 females. They were aged from 39∼72 years. The mean age was (49.65 ± 5.13) years. Inclusion criteria are as follows: being diagnosed with hepatocellular carcinoma [10] and underwent TACE; the vital signs were stable after TACE; primary school education or above; being conscious; had independent reading ability and could understand and complete questionnaires; and the patients were agreed with the study. Exclusion criteria are as follows: having no need to take TACE; survival time <3 months; having mental disease; dropping out during the study; and unable to communicate in normal language. They were divided into the control group (July 2019 to December 2019, *n* = 53) and the observation group (January 2020 to June 2020, *n* = 53) according to the admission time.

### 2.2. Method

The control group was taken care with the usual care such as renal and liver function tests, prevention of infection, and notes instruction. At the same time, intervention such as psychological counseling and scientific knowledge of health teaching was conducted on the control group.

The observation group received SFA on the basis of the control group. The SFA nursing team was composed with the head nurse, nurses who had received SFA professional education. There was one time of intervention practice for each patient, and the intervention time was 30–45 minutes. (1) Problem determination (Day 1 of admission): the basic information of the patients was obtained and it was assessed; nurse-patient communication was enhanced; the real thoughts of the patients were understood; the patient was asked whether he or she is discomfort or not; and the patients are guided to express the physical and psychological conditions, such as follows: “Do you have any problems with TACE? What are your thoughts about physical recovery? What is the quality of your recent sleep? What help would you like to receive?” Based on the results, current problems were determined. (2) Construct goals (Day 3 of admission): the patients were encouraged to construct correct and feasible goals with the medical staff; the patient was instructed on how to cooperate; and the patients were instructed to hypothesize about what benefits and changes in conditions could be achieved after the problem was managed. “What are you going to do to solve the possible complications of the TACE procedure? What methods would you use for pain relief? How do you think what you can do to improve sleep quality? If you can control diet according to doctor's advice, exercise, and improve sleep status with care, you can ease the discomfort of the procedure.” The goals were organized to guide the patients to confront the problem through communication sentences as mentioned above. (3) Explore the exception (3 days before operation): The patients were guided to carry out the plan; the patients were introduced detailed knowledge about hepatocellular carcinoma; the basic principle, treatment process, treatment effect, and precautions of TACE procedure were explained and they were helped to understand the importance of applying TACE procedure; and nurses had introduced patients to the use of analgesics and the use of analgesics at the right time to maximize the effects of pain. After the use of analgesic drugs, the occurrence of analgesic effects and adverse reaction symptoms were recorded in detail, and the patients were continuously assessed for pain. At the same time, nondrug analgesia was administered. Nursing staff guided patients to breathe deeply at a slow pace, talked to patients more, relieved their bad mood, and transferred the attention of patients. Abdominal massage was performed to relax the muscles and reduced abdominal tension to raise the pain threshold and relieved pain; distracted patients' attention through psychological suggestion, language comfort, and other measures to shift patients' attention and help them be active in fighting hepatocellular carcinoma; helped patients recall the occasional improvement; and asked “How did the pain relief happen? How can the exception continue to happen?” Through the practice mentioned above, we assisted patients to develop positive perceptions. (4) Feedback on goals (1^st^ day after operation): feedback was changed with the patient on reaching the goal with giving affirmation and support; patients were encouraged to continue the measures that work well; the methods that cannot work well were corrected; patients were encouraged with words, “With your persistence, many problems have been solved; you are now able to face the effects of the disease positively.” (5) Goal evaluation (7^th^ day after operation): the effectiveness of various aspects of complications, pain perception, sleep status, and quality of life were evaluated to encourage patients to make further efforts and to summarize and analyze the experience.

After the intervention, questionnaires were distributed to the patients and assessed by the trained research staff to observe the effects of the intervention. Researchers explained the purpose of the survey and related requirements to patients, and patients could fill in the scale with their consent. If patients could not fill in the scale in person, patients could dictate it and staff could write it for them. A total of 106 questionnaires were sent out, and 106 were effectively received with the effective recovery of 100.00%.

### 2.3. Observation Indicators

(1) Clinical data such as age, gender, classification of liver function, pathological stage, pathological type, Karnofsky Performance Status (KPS) score, and educational level were recorded for the two groups. (2) Complications such as nausea and vomiting, fever, bleeding, and renal function impairment were recorded in both groups. (3) Visual analogue scale (VAS) [11] was applied to mark the pain on a 10 cm horizontal line according to the intensity of pain which was scored from 0 to 10, with higher scores indicating stronger pain. All the measuring actions were done by the same operator. The marked points were data mined. (4) The Pittsburgh sleep quality index (PSQI) [12] was applied, with 18 entries including sleep quality, time to fall asleep, sleep duration, sleep efficiency, sleep disorders, hypnotic drugs, and daytime dysfunction. Each item was scored according to the level of 0∼3 points, and the accumulated score of each item was PSQI total score ranging from 0 to 21 points with higher scores indicating poorer sleep. Cronbach's *α* coefficient of the scale was 0.845. (5) The Generic Quality of Life Inventory-74 (GQOL-74) [13] was applied, with 74 items including physical functioning, psychological functioning, social functioning, and living status. The total score of the inventory was 100 points. The higher scores the patients got indicated the quality of their life was better. Cronbach's *α* coefficient of the scale was 0.796.

### 2.4. Statistical Methods

SPSS 22.0 software was applied for processing. The measurement data were expressed as mean ± standard deviation ($\bar{x}\pm s$), and the *t*-test was applied for comparison. The enumeration data were expressed as (%), and the *χ*^2^ test was applied for comparison. *P* < 0.05 means that the difference has statistical significance.

## 3. Results

### 3.1. Comparison of Clinical Data between the Two Groups

There was no statistically significance of difference between the two groups in the terms of age, gender, classification of liver function, pathological stage, KPS score, pathological type, and educational level (*P* > 0.05). For details, see Table 1.

### 3.2. Comparison of Complications between the Two Groups

The complication rate in the observation group (16.98%) was lower than that in the control group (33.96%), and the difference had statistical significance (*P* < 0.05). For details, see Figure 1.

### 3.3. Comparison of Pain Sensation between the Two Groups

There was no significant difference in the score of pain perception between the two groups (*P* > 0.05). For details, see Figure 2.

### 3.4. Comparison of Sleep Status between the Two Groups

All scores of sleep status in the observation group were lower than those in the control group, and the differences had statistical significance (*P* < 0.05). For details, see Figure 3.

### 3.5. Comparison of Quality of Life between the Two Groups

The observation group got higher scores of quality of life than the control group. The differences were statistically significant (*P* < 0.05). For details, see Figure 4.

## 4. Discussion

In recent years, the incidence of hepatocellular carcinoma is gradually increasing and the population is getting younger [14]. TACE is an effective clinical treatment for hepatocellular carcinoma, which can prolong patients' survival time by interrupting the blood supply to the tumor and causing tumor tissue necrosis [15, 16]. However, due to the disease progression, discomfort during the treatment, and the complications, patients undergoing TACE for hepatocellular carcinoma are prone to negative psychological conditions, which increase the patients' psychological burden and thus seriously affect their physical and mental health and the prognosis [17]. Therefore, it is necessary to adopt effective nursing means for patients undergoing TACE for hepatocellular carcinoma.

SFA is an approach that focuses on the positive aspects of the individual and discovers as much as possible his or her own potential and resources to solve the problems [18]. Karakaya's and Özgür team [19] reported that SFA plays an important role in improving self-efficacy and self-esteem levels in the adolescents with attention deficit hyperactivity disorder. Aminnasab's et al. team [20] conducted an investigation on 30 patients with breast cancer and found that the levels of depression and perceived stress of patients significantly decreased after receiving SFA intervention, so it is necessary to conduct psychological evaluation of patients with breast cancer clinically and conduct appropriate SFA intervention according to the results of the evaluation. Zhai's and Zhu team [21] conducted a survey of 120 patients undergoing vascular surgery. The results showed that after the first and second weeks of SFA, the patients had better profile of mood states scores and symptom check-list-90 scores, and the second week was better than the first week. The results suggested that SFA was beneficial to reduce negative emotions and improve the psychological state of patients.

### 4.1. SFA Can Effectively Reduce the Complications

In this study, compared with the control group (33.96%), the total incidence of complications in the observation group (16.98%) was lower. The results showed that SFA can reduce the complications in patients undergoing TACE for hepatocellular carcinoma. We speculate that the reasons are as follows: in clinical practice, traditional nursing is usually carried out for patients undergoing TACE for hepatocellular carcinoma. Although it has a certain role in nursing, it cannot mobilize the self-ability and willingness of the patients. SFA can unearth the positive power and potential of patients undergoing TACE for hepatocellular carcinoma, develop an active way of thinking, mobilize the enthusiasm for treatment, and relieve the psychological crisis. SFA can enable patients to actively participate in their own management, with the characteristics of subjectivity and enthusiasm so as to achieve the goal of positive nursing and improve the ability to prevent complications [22].

### 4.2. SFA Can Effectively Relieve Pain Sensation

We found that there was no significant difference in the score of pain perception between the two groups, but the score of pain perception in the observation group was lower than that in the control group. After summarizing many years of nursing experience, the physician in our department believes that the possible reasons are as follows: patients undergoing TACE for hepatocellular carcinoma often have varying degrees of pain sensation, which is closely related to the type and dosage of chemotherapy drugs, but nursing measures can only relieve the pain sensation to a certain extent. The SFA program focuses on introducing the knowledge of hepatocellular carcinoma in detail to patients undergoing TACE for hepatocellular carcinoma and providing adequate health education and helping them understand the importance of applying TACE surgery. At the same time, SFA can guide patients to be inspired by the excavation of motive power, causing patients to divert their attention to active anti-cancer. In addition, SFA can use a variety of ways to distract patients' attention so that patients can actively seek effective measures to reduce pain sensation and improve pain tolerance, which has a certain improvement effect. Dargan's team research reported that SFA was a method that aims to achieve patient goals by identifying and using the expertise of patients. By implementing SFA for patients with chronic pain for 8 weeks, it could relieve pain and help patients with chronic pain diseases live a good and meaningful life. Our research conclusion is roughly consistent with this conclusion [23].

### 4.3. SFA Can Effectively Improve Sleep Quality

Because patients undergoing TACE for hepatocellular carcinoma have a sense of uncertainty about the development of the disease, they are prone to a variety of adverse psychological problems, which further lead to sleep disorders such as difficulty in falling asleep, light sleep, and frequent awakening. In addition, painful stimulation may cause dysfunction of the serotonin system and its receptors, leading to rapid eye movement sleep deprivation, thereby reducing the quality of sleep in patients. The results of this study showed that the sleep of patients in the observation group was improved after the application of SFA. SFA can affect the mental health of people, increase individual enthusiasm, establish confidence in overcoming difficulties, and effectively relieve bad emotions. In addition, SFA can reduce the level of pain sensation, thereby reducing the stimulation to the patient and improving the quality of sleep in patients [24].

### 4.4. SFA Can Effectively Improve the Quality of Life

SFA can guide patients to actively look for problems, formulate scientifically feasible goals, explore practices where exceptions occur, listen to feedback, summarize and evaluate, and divert patients' attention to solutions to problems. The SFA model provides health education to patients according to their existing problems, stimulates their subjective initiative, and encourages patients to discover their own progress. And it can enhance the confidence in fighting the disease so that makes patients realize their self-worth, fully mobilize the enthusiasm for life, and reduce the idea of avoiding and succumbing so as to eliminating difficulties and problems and improve the standard of living. We found that the observation group had a higher quality of life scores, which suggests that SFA can improve the quality of life of patients undergoing TACE for hepatocellular carcinoma [25].

## 5. Conclusion

In conclusion, SFA can effectively reduce the complications, relieve pain, improve sleep quality, and improve the quality of life in patients undergoing TACE for hepatocellular carcinoma and is worthy of clinical application. With the transformation of medical mode and the improvement of people's living standards, patients have more demands for comfort during hospitalization. Through the application of SFA, it proves that as long as medical staff have a high sense of responsibility and focus on the patients and do a good job of nursing from the details, they will be able to meet the health needs of patients.

However, it should be noted that the number of selected cases in this study is small and only evaluated the patients' nursing efficiency in a short period of time. Therefore, it is still necessary to carry out a large sample and long-term investigation in future studies, which will also become the focus of our team's future research.

## Figures and Tables

**Figure 1:** Comparison of complications between the two groups. Note: compared with the control group, ^*∗*^*P* < 0.05.

**Figure 2:** Comparison of pain sensation between the two groups.

**Figure 3:** Comparison of sleep status between the two groups. Note: compared with the control group, ^*∗*^*P* < 0.05.

**Figure 4:** Comparison of quality of life between the two groups. Note: compared with the control group, ^*∗*^*P* < 0.05.

**Table 1:** Comparison of clinical data between the two groups (*n*, $\bar{x}\pm s$, %).

Group	Age (years)	Gender		Classification of liver function		Pathological stage		Pathological type		KPS score (points)	Educational level		
		Male	Female	Grade A	Grade B	I∼II	III∼IV	Unicellular carcinoma	Carcinoma		Elementary school	Junior high school	High school and above
Control group (*n* = 53)	49.28 ± 7.50	31 (58.49%)	22 (41.51%)	40 (75.47%)	13 (24.53%)	29 (54.72%)	24 (45.28%)	36 (67.92%)	17 (32.08%)	72.65 ± 8.19	16 (30.19%)	23 (43.40%)	14 (26.42%)
Observation group (*n* = 53)	50.03 ± 7.69	29 (54.72%)	24 (45.28%)	41 (77.36%)	12 (22.64%)	30 (56.60%)	23 (43.40%)	34 (64.15%)	19 (35.85%)	74.02 ± 7.86	18 (33.96%)	20 (37.74%)	15 (28.30%)
*t*/*χ*^2^-value	0.508	0.153		0.052		0.038		0.168		0.878	0.361		
*P* value	0.612	0.695		0.819		0.844		0.682		0.381	0.835		

## Data Availability

The data that are used or analyzed in the research can be obtained from the corresponding author upon reasonable request.
